# Nonmedical Determinants of Congenital Heart Diseases in Children from the Perspective of Mothers: A Qualitative Study in Iran

**DOI:** 10.1155/2021/6647260

**Published:** 2021-08-17

**Authors:** Maryam Borjali, Mostafa Amini-Rarani, Mehdi Nosratabadi

**Affiliations:** ^1^Department of Health and Social Welfare, School of Management and Medical Information Sciences, Isfahan University of Medical Sciences, Isfahan, Iran; ^2^Health Management and Economics Research Center, Isfahan University of Medical Sciences, Isfahan, Iran; ^3^Social Determinants of Health Research Center, Isfahan University of Medical Sciences, Isfahan, Iran

## Abstract

**Introduction:**

Mortality due to noncommunicable diseases has increased in the world today with the advent of demographic shifts, growing age, and lifestyle patterns in the world, which have been affected by economic and social crises. Congenital heart defects are one of the forms of diseases that have raised infant mortality worldwide. The objective of present study was to identify nonmedical determinants related to this abnormality from the mother's perspectives.

**Methods:**

This research was a qualitative study and the data collection method was a semistructured interview with mothers who had children with congenital heart diseases referring to the Shahid Rajaei Heart Hospital in Tehran, Iran. A thematic analysis approach was employed to analyze transcribed documents assisted by MAXQDA Plus version 12.

**Results:**

Four general themes and ten subthemes including social contexts (social harms, social interactions, and social necessities), psychological contexts (mood disorders and mental well-being), cultural contexts (unhealthy lifestyle, family culture, and poor parental health behaviors), and environmental contexts (living area and polluted air) were extracted from interviews with mothers of children with congenital heart diseases.

**Conclusions:**

Results suggest that factors such as childhood poverty, lack of parental awareness of congenital diseases, lack of proper nutrition and health facilities, education, and lack of medical supervision during pregnancy were most related with the birth of children with congenital heart disease from mothers' prospective. In this regard, targeted and intersectorial collaborations are proposed to address nonmedical determinants related to the incidence of congenital heart diseases.

## 1. Introduction

Health viewpoints have gained a wider outlook in today's world and particular attention has been paid to nonmedical determinants of health. Nonmedical determinants, such as lifestyle behaviors, environment conditions, and socioeconomic status affect and cause inequities in the health condition, including quality of life [1, 2]. It is true that medical care can extend the life or treatment of serious illness, but the social, economic, and environmental circumstances that make people sick or in need of care are crucial for the health of the community. [3].

Congenital anomalies are considered one of the leading causes of death and one of the leading causes of disability, accounting for 10% of deaths in children under the age of 5 [4]. Birth and care of a fetus and then a baby with abnormalities have adverse effects on the physical, psychological, social, and economic aspects of the family [5, 6].

Congenital heart diseases (CHD) are one of the most common disordered congenital disorders in the field of community health. During fetal development, these anomalies occur and affect the newborn from birth and are among the most common birth defects, causing death in infancy and childhood [7, 8]. The incidence of this disease is approximately 6 to 8 cases per 1000 live births [9, 10]. The etiology of most congenital heart defects is unknown. Studies have shown that, due to the complex combination of environmental teratogens and social and genetic factors, approximately 50 to 85 percent are involved in the development of this disease [11, 12]. Studies conducted in Iran have estimated the prevalence of congenital heart abnormalities in the range of 9.7 to 17.5 per 1000 live births [13, 14].

Nonmedical determinants, including cultural, environmental, and social determinants of health have a significant impact on the incidence and prevalence of congenital heart defects [11]. Nonmedical determinants during life affect the health of people in society and are one of the foundations of lifestyle choices in society, including the lives of pregnant mothers [15]. In other words, the incidence and prevalence of congenital heart disease are strongly influenced by these nonmedical determinants [10, 16].

In recent years, nonmedical health determinants have been shown to contribute to health and disease outcomes and lead to congenital anomalies [17, 18]. Poverty, social exclusion, and unhealthy behaviors are associated with congenital anomalies such as congenital heart abnormalities, although in this regard, the results of research are different [10]. Moreover, the results of epidemiological studies show the adverse effects of environmental pollutants on fetal health and growth [19] and this case has been mentioned in studies on congenital CHD [20].

By identifying nonmedical determinants from the perspective of mothers having children with CHD, it is possible to explore the sociocultural background in which these women were born, grew up, and lived and the role that such a context plays in the knowledge, health habits, and ultimately the development of congenital heart disease in children. On the other hand, social and environmental contexts can also determine the quality of maternal care during pregnancy [21]. Mothers are also unaware of the consequences of some of the complications that arise during or before pregnancy that contribute to some heart problems and disorders for the infant. [22]. By identifying the perspectives of mothers who have children with CHD, it is possible to find out in which society these mothers decided to become pregnant and what the level of maternal care was during pregnancy and how availability is to healthcare in the community which these mothers live. Therefore, improving sociocultural contexts is one of the priorities to prevent the occurrence and spread of CHD, since these contexts can shape mothers' pregnancy behaviors.

In view of the variety of unfavorable sociocultural contexts and, on the other hand, environmental risk factors such as air pollution and biochemical substances in Iran, as predisposing factors for CHD, it is important to carry out studies to identify precisely such nonmedical determinants [7, 23]. Considering that no research has been conducted in this field in Iran, the present study seeks to identify the views of mothers who have children with CHD in the field of nonmedical factors linked to this disease in order to provide the basis for causal studies.

## 2. Method

### 2.1. Design and Setting

This study was a qualitative study that was designed with a thematic content analysis approach to identify nonmedical determinants of CHD from the perspective of mothers. The temporal realm of the present study in 2019 and the setting was Shahid Rajaee Cardiovascular Center in Tehran, Iran. This center is one of the largest heart hospitals in Asia. This hospital was founded in 1974. At present, it has more than 600 active beds and receives about 1000 patients daily from different parts of Iran.

### 2.2. Data Collection

In this study, data were collected through semistructured interviews. First, the interview guide was prepared based on the objectives of the research. Purposeful sampling was performed among mothers having children with CHD who referred to Shahid Rajaei Cardiovascular Center in Tehran. After selecting the interviewee, the purpose of the interview was explained and after obtaining the verbal consent, the face-to-face interview was performed according to the guide prepared by one research team (MB). Data collection continued until reaching the saturation point. In interview 20, the data was saturated and subsequent interviews were stopped.

Each interview lasted between 30 and 90 minutes, all interviews were recorded, and important points and events were recorded during the interview. A general question was first asked, “How did your life go from childhood to the birth of your child with CHD?” Other exploratory questions were then asked based on the mother's response.

### 2.3. Data Analysis

Data analysis was performed using thematic analysis approach (explicit and implicit content). The six-step process proposed by Braun and Clarke [24] was used to perform thematic analysis as follows.

According to the first step, two researchers (MB and MN) became familiarized with the data through listening to the recorded interviews and repeated reading of the transcribed data. Also, MB and MN actively searched for meanings and underlying patterns of data.

At second stage, the researchers generated the initial codes from the original data and the most related segments were identified and attached to each code (i.e., coded segments created). After all the data were primarily coded and coded segments identified, we organized and summarized the initial code in order to achieve a general theme. Also, subthemes within themes were found. In forth stage, the extracted themes and subthemes were read, re-read, and discussed during three two-hour sessions with the members of the research team. At this stage disagreements resolved and consensus was reached between the researchers in terms of themes, subthemes, and codes. At fifth stage, the overlap between themes and subthemes was carefully examined, definition of themes was finalized, and final names were given to the themes and subthemes. Eventually, the scholarly article that resulted from the analysis was wrote up.

### 2.4. Trustworthiness Criteria

To evaluate the quality of the present study, four criteria were used: credibility, transferability, dependability, and conformability proposed by Lincoln Goba [25].

To ensure the credibility of the data, in addition to the researchers' prolonged engagement with a study of about 13 months, mothers were selected who had enough experience living with a child with CHD. For transferability of the findings, appropriate study samples were purposefully selected and data collection and analysis were performed simultaneously. Direct citations were also used in the text and a rich description of the data was provided in this study.

Dependability was performed through cross-checking with the cooperation of an external auditor. In this regard, contradictory and negative cases were examined to investigate the reasons for this discrepancy in the findings, and then the supplementary opinions of the research team, under the supervision of an external consultant, were summarized and after agreeing the text was coded and analyzed and the findings were modified.

In order to increase the conformability, it was tried not to interfere with individual values and theoretical orientations of the research team in the research process and extract the findings by observing the neutrality of the researchers.

### 2.5. Findings

Characteristics of interviewee are described in Table 1. Mothers were on average 25 years old and mostly graduated from under diploma. Moreover, interviewees' husbands mostly were under diploma and occupied in worker jobs.

Four main themes and 10 subthemes were extracted from interviews regarding nonmedical determinants of CHD in children from the mothers' perspective. The themes were social contexts, psychological contexts, cultural contexts, and environmental contexts.

Figure 1 shows extracted themes and subthemes. Also, Table 2 shows codes corresponding to each subtheme.

### 2.6. Social Contexts

#### 2.6.1. Social Harms

This subtheme discusses the cases and concerns that a family will suffer from in a potentially unhealthy society and cope with the resulting complications and injuries. Categories such as seasonal father unemployment, maternal work from childhood, using of alcohol and tobacco by parents, gender discrimination, and poverty during pregnancy were among the social harms mentioned in interviews with mothers.

In this regard, an interviewee stated:
    “My husband is unemployed and addicted, he does not work and sometimes he does not come home at all. He leaves me and the children left alone. He has not paid any money to his family for 3 years and is just following for her addiction.” (Interviewee number 13).

Or another interviewee mentioned poverty during pregnancy:
    “I had a stressful and poor pregnancy and we also had problems with my livelihood. Due to the poverty, I was not able to see a doctor and I was not taken care of. I had poor nutrition because of my poor financial situation and I could not use proper food. We had a hard time paying our rent.” (Interviewee number 17).

#### 2.6.2. Social Interactions

This subtheme consisted mostly of codes that referred to social interactions between mother, family, and community, each of which could in some way be related to the childbearing with a CHD, with issues such as the mother's social isolation, weak social networks, and social exclusion due to immigration. In this regard one of the interviewees noted the following:

“My husband is addicted, and our family is excluded by others because of a lot of issues, and others don't come and go with us because of my husband's addiction. Since we're poor, and my husband is like that, the neighbors don't come and go with us a lot. My children and I have almost no contact with anyone and it is very difficult for us.” (Interviewee number 13).

When a family migrates, they move away from their native family, resulting in inconsistencies in their social interactions with the new community environment that can be problematic for the family. In the field of immigration, one interviewee stated the following:

“When I got married, we migrated from the villages of Ardabil to the around of Tehran. We have no interaction with anyone here.” (Interviewee number 19).

#### 2.6.3. Social Requirements

In this subtheme, codes were extracted that referred to the needs, requirements, and social needs. These topics can include the needs and facilities that the community should provide for the family or the needs that the family and the community should provide for the mother, such as appropriate educational facilities, appropriate health facilities, and medical treatment.

  In this regard an interviewee mentioned the following:
  “I was born in the villages of Sistan and Baluchestan and due to the lack of educational facilities, children dropping out of school, especially girls, because they cannot go to other villages to continue their education.” (Interviewee number 5).
  Or an interviewee referred to the field of health facilities:
  “My husband and I have thalassemia minor and we got married without any information. I used to go to the health center before I got pregnant and they did not give me any information about pre-pregnancy genetic testing. There was no doctor in the health center and the staff told me not to follow the fetus situation because you are annoying yourself and it is useless and they gave me wrong advice.” (Interviewee number 12).

### 2.7. Psychological Contexts

Subthemes and codes relevant to the psychological health of families and mothers in society and its challenges and implications in terms of childbearing with CHD have been included in this theme, such as mother's distress, maternal frustrations from childhood, drug use by father due to mood disorders, and lack of emotional support by mother.

  Regarding the mother's mood disorder, an interviewee mentioned the following:
  “I was in the Bam city and I lost my family in the earthquake and was very dysthymia. I went to the doctor who told me that I have a severe mood problem and I need to be treated by a psychiatrist. I was also much agitated during pregnancy because my wife and I had thalassemia.” (Interviewee number 13).
  Another interviewee noted the unfavorable psychological conditions in childhood and stated the following:
  “Because we lived in war zones, we suffered a lot of anxiety and fear as children. The cultural pressures in our lives and early marriage put a lot of stress on me.” (Interviewee number 10).

### 2.8. Cultural Contexts

#### 2.8.1. Unhealthy Lifestyle

The subthemes were related to some issues such as type of pregnancy and the parents' illnesses, their age and their way of dealing with congenital anomalies, and, in general, the issues of mistakes and wrong methods in people's lifestyles.

  An interviewee referred to an unwanted pregnancy:
  “We had a poor life and I was not under the care of a doctor and I did not know I was pregnant. When I got pregnant, I did not have the necessary pregnancy tests.” (Interviewee number 18).
  Or an interviewee referred to the field of noncompliance to the medical measures:
  “I did not follow up much during my pregnancy and only went to a midwife twice because I did not think my baby might be born ill.” (Interviewee number 20).

#### 2.8.2. Family Culture

This subtheme refers to the marriage and related issues, the culture of childbearing and consanguineous marriage, the population of families and relatives and their culture, and the discriminatory and traditional view of the role of women in the family.

  Regarding violence to childbearing, one interviewee mentioned the following:
  “Because my husband's brother did not have children, my husband's family pressured me to have children.” (Interviewee number 9).
  Or regarding humiliating and traditional view of the role of women in the family and society, an interviewee mentioned the following:
  “Because childbearing is very important in our place of residence and in our family culture, and if I do not have a child for any reason, the family will see it through my eyes and my wife will leave and divorce me.” (Interviewee number 6).

#### 2.8.3. Improper Parental Health Behaviors

This subtheme refers to the behaviors and actions of parents that are related to congenital anomalies. Items such as lack of timely information about the child's illness, lack of following up and treatment of former congenital anomalies, and maternal pregnancy after abortion.

  An interviewee referred to the former congenital anomalies of the children in the family:
  “Each of my children is somehow sick, even though my first child was ill, but no one took him to the doctor and my husband did not pay attention until this third child was born unintentionally with a heart problem.” (Interviewee number 14).
  Or another interviewee mentioned the following regarding postabortion pregnancy:
  “I became pregnant four times and my first and third children were aborted. I do not know the reason for my abortions and I did not go to the doctor for follow-up. I continued to childbearing without the necessary care.” (Interviewee number 12).

### 2.9. Environmental Contexts

This theme refers to issues that existed naturally in a person's living environment and the person could have been affected by them. In the meantime, polluted climates, fine dust, and extreme heat were the issues most frequently mentioned in interviews.

#### 2.9.1. Living Area

In a number of interviews, the exhausting warmth of the living environment has been mentioned. On the other hand, some have migrated to a place where they had to endure very hot weather.

  An interviewee noted:
  “Our place of residence is in Ahvaz, the air has been polluted for years due to dust, and in some seasons it is difficult to breathe.” (Interviewee number 1).

#### 2.9.2. Polluted Air

In some interviews, the issue of polluted air is mentioned. The mother has lived in that place in the time of the mother's childhood to the marriage, pregnancy, and delivery of the sick child. This can affect the fetus and baby just like taking illicit drugs during pregnancy.

  An interviewee noted:
  “There is air pollution in my living area because there are factories around that pollute the air.” (Interviewee number 2).

## 3. Discussion

The present study identified nonmedical determinants of CHD from the perspective of mothers in Iran. Four themes including social, psychological, cultural, and environmental contexts were extracted from the interviews. The theme of social contexts included three subthemes of social harms, social interactions, and social necessities. A study conducted by Xiangi et al. which examined the socioeconomic status and risk of congenital heart disease in infants in China found that the economic and social status of mothers, mothers' education, and family income affect the birth of infants with CHD [26]. The study by Zimmerman and Sable revealed that being born and growing up in poverty and poor conditions increases the risk of heart disease and children born into poor families are more prone to CHD and chronic diseases [27].

Our research also showed, in the theme of social necessities, factors such as educational, health, and food poverty, as indicators of low socioeconomic status of mothers [26, 28]. In addition, maternal poverty from childhood was associated with the birth of a child with CHD. In this regard, and in line with our findings, a case-control study on pregnant women showed that pregnant mothers who were nutritionally better during and before pregnancy and had a better dairy diet pattern, compared to the control group, and were at lower risk of having an infant with CHD [29]. Along with the findings from the interviews in our study, other studies have shown that family poverty from childhood is associated with the birth of infant with CHD [30, 31].

Based on the findings extracted from interviews, mothers stated low social interactions and thus limited access to social networks. It seems that these deficiencies can play a role in the development and spread of CHD in children through mechanisms such as causing anxiety [32], inadequate access to care-preventive centers [33], and the lack of emotional-informational support [34]. Consistent with our results, a ten-year literature review showed that lack of social communication and low social support are considered as risk factors for diagnosing heart disorders [35].

Social exclusion due to migration was mentioned in interviews with mothers as one of the concepts related to CHD. It seems that immigration is effective in the incidence of congenital heart disease through mechanisms such as unemployment, lack of appropriate facilities, social isolation, lack of financial and emotional support, poverty, and financial problems. Studies in this regard also revealed that migration from the homeland can increase the risk of exposure to risk factors for cardiovascular disease (in the terms of harmful food consumption, obesity, smoking, etc.) [36, 37].

A study conducted by Ahmadi et al. [37] on children with CHD and healthy children in Iran showed that the history of alcohol and tobacco use during pregnancy has had an impact on the birth of children with heart disease and children whose mothers smoked were 5 times more likely to develop CVD than healthy group. In our study, under the subtheme of social harms, items such as alcohol and smoking in the families of children with CHD were extracted. In this regard, a meta-analysis study showed that maternal alcohol consumption during pregnancy was strongly associated with the incidence of CHD [38]. Another study showed an association between exposure to tobacco smoke and the incidence of CHD in the child [39]. It has been shown that using of alcohol and tobacco by the father is significantly associated with the risk of congenital heart disease in children [40, 41]. Possible explanations and mechanisms for this relationship include that the father's exposure to alcohol can alter DNA methylation in sperm, which significantly reduces the activity of DNA transferase enzyme, followed by gene silencing, and it results in congenital anomalies in children [41, 42]. This finding indicates that raising health awareness in parents is necessary to prevent exposure to alcohol and tobacco before, during, and after pregnancy.

In the theme of mental contexts, two subthemes of mental illness and mental well-being were extracted. Numerous studies have shown that parents, especially mothers of children with CHD, have more mental health problems (such as depression, anxiety, and guilt) and more sociopsychological adjustment problems than parents with healthy children or children with other medical problems [43, 44]. It has been reported that these disorders can lead to a number of mental-psychological conflicts, which in turn affect preventive measures and care to diagnose the disease before and after pregnancy [45, 46].

Parents' mental health problems can exist in different stages of children's lives and their medical processes. A recent systematic study found that up to 30% of parents of children with CVD have symptoms of posttraumatic stress disorder (PTS), 25–50% of them report symptoms of depression or anxiety, and 30 to 80% report severe mental anxiety [47]. In addition, after heart surgery for children, parents have to face various physical, financial, and other practical challenges.

The third main theme extracted from the interviews with mothers was cultural contexts.

In this theme, three subthemes including unhealthy lifestyle consequences, family culture, and incorrect health behaviors of parents were identified, and factors such as lack of timely information about the child's illness, lack of following up of congenital anomalies, unwanted pregnancy, and consanguineous marriage in the interviews were mentioned. Heart disorders are problems that occur before birth, during pregnancy, and during the formation of the fetal heart and important lifestyle and behavioral characteristics of parents, especially mothers, affect the development of this disease [48]. Our study on CHD showed that the living conditions of mothers from childhood to pregnancy and childbirth affect the health of the child (especially heart health). Siabani and colleagues in a systematic review study emphasized on the important role of cultural and lifestyle factors in the occurrence of CHD in different provinces of Iran. Indeed, their research has shown that some people are more likely to cause children to develop congenital heart disease due to hereditary background or improper lifestyles. Knowing the risk factors for these diseases will therefore help individuals to prevent CHD [49].

From the findings of the interviews of the present study, it can be inferred that cultural factors such as large families, disregard for medical measures, and indifference to congenital disorders in the family can lead to CHD in children. For example, families with low facilities and large family sizes may be subjected to cultural poverty, lack of adequate nutrition and health facilities, and lack of mental well-being, which may contribute to ignorance about healthcare and disease prevention.

Along with our study, other research has shown that cultural issues, including the consequences of an unhealthy\ lifestyle, are important in CHD. Mothers who often had unwanted pregnancies and used various drugs during pregnancy were at higher risk of giving birth to children with CHD [50, 51]. According to the findings, the lifestyle of mothers with CHD children was far from health awareness, and going to a doctor or following medical measures was not important for them. These mothers often became pregnant without any prepregnancy preparations and were unaware of the existence of prepregnancy preparations. These mothers were indifferent to congenital disorders in their other children or children of close relatives due to lack of information or lack of consultation with the doctor prior to pregnancy.

The fourth theme obtained from interviews with mothers with CHD children was environmental contexts such as hot climates and air pollution. In our study, some mothers reported being exposed to extreme heat and air pollution during their pregnancies. In a case-control study by Davand et al. [52] maternal exposure to air pollution has been shown to be associated with a wide range of adverse pregnancy outcomes, such as CHD. In our study, it was found that the living environment of some mothers was air polluted. This condition is very important for pregnant women because the fetus is also affected by these factors. In a study conducted by Zang et al. which examined mothers' exposure to heat in early pregnancy and its effect on congenital heart disease, it was found that congenital heart defects are more common in the summer [53]. Heat appears to have an impact directly or with other modulators on a heat stress response. Some studies have shown that exposure to high temperatures can lead to cell death in the fetus and subsequent congenital heart defects [54].

In the field of air pollution, which was another code extracted in the present study, studies have shown that air pollution is associated with CHD children [55, 56]. These findings suggest that oxidative stress caused by air pollution during early pregnancy may affect heart development. However, the periods of vulnerability to these environmental pollution-related side effects may not directly correspond with the stages of fetal heart growing.

## 4. Conclusion

In general, the study showed that social, psychological, and cultural determinants such as childhood poverty, inadequate education, lack of proper nutrition, poor lifestyle patterns, parents' ignorance of consanguineous marriages, and congenital disorders, as well as environmental factors such as heat and the presence of dust and air pollution, can be considered as contexts that contribute to the occurrence, spread, and complications of CHD. Investing in socioeconomic status, improving social facilities and necessities, and raising household awareness regarding the social, cultural, and environmental risk factors associated with congenital heart disease can be beneficial. Intersectorial collaborations which address nonmedical determinants of health should also be adopted to reduce the risk factors associated with the birth of children with CHD.

## Figures and Tables

**Figure 1:** Themes and subthemes related to the birth of child with CHD from the mothers' perspective.

**Table 1:** Characteristics of interviewed mothers.

Interviewee number	Age	Education level	Husband's occupation	Husband's education level
1	27	Diploma	Nonclerical job	Middle school
2	31	Middle school	Worker	Illiterate
3	17	Illiterate	Nonclerical job	Illiterate
4	41	Illiterate	Unemployed	Illiterate
5	20	Primary school	Unemployed	Illiterate
6	19	Primary school	Worker	Primary school
7	21	Illiterate	Unemployed	Middle school
8	25	High school	Driver	Middle school
9	20	Diploma	Police officer	Diploma
10	22	Illiterate	Worker	Illiterate
11	28	Diploma	Worker	Middle school
12	36	Primary school	Unemployed	Illiterate
13	18	Illiterate	Unemployed	Illiterate
14	46	Diploma	Farmer	Primary school
15	30	Illiterate	Worker	Illiterate
16	27	Diploma	Worker	Middle school
17	18	Middle school	Unemployed	Middle school
18	15	Primary school	Driver	Primary school
19	28	Middle school	Worker	Middle school
20	18	Diploma	Worker	Middle school

**Table 2:** Themes (categories), subcategories, and codes related to nonmedical determinants associated with CHD in children based on mothers' perspectives.

Theme	Subtheme	Codes
Social contexts	Social harms	Father's seasonal unemployment
		Poverty of the mother's family since childhood
		Family poverty
		Father alcohol consumption
		Drug in parent families
		Father's tobacco consumption
		Father's smoking
		Gender discrimination
		Working mother since childhood
	Social interactions	Maternal social isolation
		Poor social networks
		Social exclusion due to migration
	Social necessities	Lack of access to appropriate educational facilities
		Lack of proper health, treatment, and medical facilities
		Lack of proper nutrition facilities

*Psychological contexts*	Mood disorders	Mother's distress
		Feeling of agitation
		Dysthymia and frustration
	Mental well-being	Lack of mental peace of the mother since childhood
		Deprivation of emotional support in mother

*Cultural contexts*	Unhealthy lifestyle	Nonuse of contraception which leads to unwanted pregnancy
		Improper use of drugs
		Disregard to medical measures
		Childbearing without background knowledge
		Indifference to the existence of congenital disorders in families
	Family culture	Forced childbearing
		Mother's second marriage
		Parental consanguineous marriage
		Kinship marriage of relatives
		Prevent of education
		Crowded family
		Humiliation of woman in the family
	Improper parental health behaviors	Maternal pregnancy after abortion
		Lack of timely information about the child's illness
		Lack of following up and treatment of former congenital anomalies

*Environmental contexts*	Living area	Very hot weather in the living area
		Crowded neighborhood
	Polluted air	Lack of safe drinking water
		The presence of dust in the air
		Dusty air

## Data Availability

The data are available on request due to privacy/ethical restrictions.
